# High efficiency wide gap Cu(In,Ga)Se_2_ solar cells: Influence of buffer layer characteristics

**DOI:** 10.1016/j.heliyon.2024.e36965

**Published:** 2024-08-27

**Authors:** Shiqing Cheng

**Affiliations:** College of Physics and Electronic Science, Shanxi Datong University, Shanxi, 037009, China

**Keywords:** Thin film solar cells, CIGS, Wide bandgap, Interfacial recombination, High efficiency

## Abstract

Wide-gap Cu(In,Ga)Se_2_ (CIGS) solar cells exhibit a superior match to the solar spectrum, resulting in a higher ideal efficiency (*E*_ff_). However, in reality, their device *E*_ff_ is lower than that of narrow-gap CIGS solar cells. This study aims to identify the factors that limit the performance enhancement of wide-gap CIGS solar cells, focusing on the characteristics of the buffer layer. The influence of the thickness and doping concentration of the CdS layer on the built-in electric field and interfacial recombination of the heterojunction has been investigated through simulation. The simulation results indicate that when the doping concentration of the CdS layer is lower than or similar to that of the CGS layer, decreasing the thickness of the CdS layer (e.g., 10 nm) is beneficial for improving device performance. However, if it is higher than that of the CGS layer, increasing the thickness of the CdS layer (e.g., 50 nm) is conducive to improving device performance. The thickness of the CdS layer that maximizes the *E*_ff_ of the wide-gap CGS device should be approximately 50 nm, and its doping concentration should be higher than that of the CGS layer. This optimization can simultaneously enhance the built-in electric field of the heterojunction and minimize its interfacial recombination, thereby improving the open-circuit voltage and *E*_ff_ of wide-gap CGS devices.

## Highlights

• Buffer properties impact built-in electric field and recombination in CGS solar cells.
• Lowering CdS thickness boosts *η* when doping content is low or similar to CGS layer's.
• Increasing CdS thickness boosts *η* when doping content surpasses the CGS layer's level.

## 1 Introduction

In recent years, CIGS thin-film solar cells have been widely used in large-scale industrial production. Ideal terrestrial solar cells should have a wide bandgap of 1.5 eV or higher to match the solar spectrum [[1], [2], [3]]. Therefore, in the case of CIGS solar cells, their absorber should have a high Ga/(Ga + In) ratio (GGI ≥0.8) to achieve a bandgap of 1.5 eV. In addition to their high ideal efficiency (*E*_ff_), wide-gap CIGS solar cells exhibit high open-circuit voltage (*V*_OC_), low short-circuit current density (*J*_SC_), and an optimal temperature coefficient. These features are beneficial for reducing losses caused by the interconnection between individual cells, making them more suitable for large-area modules. Moreover, wide-gap CIGS solar cells are suitable for space applications owing to their strong antiradiation abilities, which can effectively help reduce *V*_OC_ losses in space devices. However, in reality, CIGS solar cells with a narrow bandgap (1.15–1.2 eV) and a GGI of 0.3–0.4 are the most efficient [[4], [5], [6], [7], [8], [9]]. The main reasons for the low *E*_ff_ of wide-bandgap CIGS solar cells are (1) high deep-level defect concentration [1,10] and low carrier collection [11] and (2) high interfacial [[12], [13], [14]] and bulk recombination [15,16], which limits the increase in the *V*_OC_ of devices. Therefore, the performance of wide-bandgap CIGS solar cells needs to be improved considerably. Setareh et al. used KF-PDT to enhance carrier collection and reduce CIGS/CdS heterojunction interfacial recombination, thereby increasing *V*_OC_, *J*_SC_, and *E*_ff_ of wide-bandgap CIGS solar cells [17]. Miguel et al. improved the grain boundary properties of wide-bandgap CIGS films by increasing the substrate temperature to 600°C-650 °C. Using this approach, they reduced the recombination loss of the absorber, thereby improving the *V*_OC_ and *E*_ff_ of the CIGS device [18]. Kanevce et al. proposed that the surface inversion of the wide-bandgap CIGS absorber could help improve device performance [12]. Larsson et al. used the adjustable bandgap Zn_1−x_Sn_x_O_y_ buffer layer to match the bandgap with a CGS thin film, thereby considerably improving the *V*_OC_ and performance of CGS devices [19]. Moustafa et al. used an adjustable bandgap ZrS_x_Se_2−x_ buffer layer and MoSe_2_ interfacial layer to improve the performance of CIGS solar cells [[20], [21], [22]]. The aforementioned approaches help improve the performance of wide-bandgap CIGS solar cells by adjusting absorber characteristics (i.e., by changing surface characteristics or grain boundary characteristics) or improving the bandgap matching of heterojunctions. However, few studies have been conducted to improve the *E*_ff_ of devices by simultaneously enhancing the built-in electric field and reducing interfacial recombination. Therefore, this study focuses on how to adjust buffer characteristics to address the aforementioned problem. We use wide-gap CGS cells to investigate the influence of CdS buffer layers with different doping concentrations and thicknesses on the built-in electric field and recombination of wide-bandgap CIGS solar cells [23]. Thus, we can identify the optimal thickness and doping concentration of the CdS film, which can enhance the built-in electric field of the heterojunction and minimize its interfacial recombination, thereby improving the performance of CGS solar cells. Simulation results indicate that for wide-gap CGS thin-film solar cells, when the CdS film doping concentration is lower or similar to that of the CGS thin film, decreasing the thickness of the CdS film (e.g., 10 nm) is beneficial to improving CGS device performance. However, when the doping concentration of the CdS film is higher than that of CGS film, increasing the thickness of the CdS film (e.g., 50 nm) to a certain extent can help improve the performance of CGS devices. To maximize the performance of CGS devices, the doping concentration of CdS thin films should be higher than that of CGS thin films, while increasing the thicknesses of the CdS thin films accordingly.

## 2 Methods: simulation

Herein, the SCAPS simulation software [24,25] is used to analyze the effects of thickness and doping concentration of the CdS layer on the performance of CGS devices. This analysis focuses on two aspects. First, the effect of the CdS film thickness on the built-in electric field and the recombination of CGS devices is studied. Second, the effect of doping concentrations of CdS films on the built-in electric field and the recombination of CGS devices is investigated. The thicknesses and doping concentrations (*N*_D_) of the CdS films range from 10 to 100 nm and 10^15^–10^17^ cm^−3^, respectively. The doping concentration of the CGS absorber (*N*_A_) is 10^16^ cm^−3^. The interface defects of the CGS/CdS interface are neutral, with electron and hole capture cross sections of 10^−13^ cm^−2^. The distribution of interface defects is single, with a total defect density of 10^12^ cm^−2^. The interface defect energy level (*E*_t_) is located 0.8 eV above *E*_V_, with electron and hole interface recombination rates (*S*_n_/*S*_p_) of 10^6^/s. Moreover, the defects of the films in the simulation are neutral, with a defect density of 10^14^ cm^−3^. The defect energy level *E*_t_ is located 0.6 eV above *E*_V_. The other parameters of the simulation are listed in Table 1. The absorption coefficient curves of the materials used in the simulation are depicted in Fig. S1, sourced from internal SCAPS data.

**Table 1:** Material parameters used in simulation [23,[26], [27], [28]].

Layer	window	window	Buffer	Absorber
parameter	Al-ZnO	i-ZnO	CdS	CGS
*E*_g_ (eV)	3.5	3.5	2.4	1.68
*N*_D_ (cm^−3^)	10^18^	10^16^	10^15^,10^16^,10^17^	10^16^
*χ* (eV)	4.42	4.42	4.2	3.68
Thickness(nm)	350	50	10,30,50,100	2000
ε/ε_0_	10	10	10	13.6
*N*_C_[cm^−3^]	1 × 10^18^	1 × 10^18^	1 × 10^18^	1 × 10^18^
*N*_V_[cm^−3^]	1 × 10^19^	1 × 10^19^	1 × 10^19^	1.8 × 10^19^
*μ*_n_[cm^2^/(Vs)]	100	100	100	100
*μ*_p_[cm^2^/(Vs)]	25	25	25	25
υ_tn_[cm/s]	1 × 10^7^	1 × 10^7^	1 × 10^7^	1 × 10^7^
υ_tp_[cm/s]	1 × 10^7^	1 × 10^7^	1 × 10^7^	1 × 10^7^

## 3 Effect of CdS layer characteristic on the performance of CGS devices

### 3.1 Effect of CdS layer thickness on the performance of CGS devices

Fig. 1a shows the band diagram of CGS solar cells with CdS layer doping concentrations of 10^15^–10^17^ cm^−3^ and thicknesses of 10–100 nm. According to Fig. 1a–c and equation (1) [29], when the doping concentration of the CdS film is confirmed (i.e., 10^15^–10^17^ cm^−3^), the built-in electric field *V*_bi_ of CGS solar cells increases with an increase in the thickness of the CdS film. This approach is beneficial for improving the *V*_OC_ of the device (Fig. 1a).

$${qV}_{\text{bi}}=E_{g,a}-E_{p,a}-E_{n,w}+{\Delta E}_{C}^{a,b}+{\Delta E}_{C}^{b,w}\ldots \ldots \ldots \ldots \ldots \ldots \ldots \ldots \left(1\right)\left[29\right]$$

(*E*_g,a_ is the energy band of CGS absorber, *E*_p,a_ is the difference between Fermi level *E*_f_ and *E*_V,CGS_, *E*_n,w_ is the difference between *E*_c,w_ (bulk) and *E*_f_, $\Delta E_{c}^{a,b}=\chi_{\text{CGS}}-\chi_{\text{CdS}}$, $\Delta E_{C}^{b,w}=\chi_{\text{CdS}}$-$\chi_{i-\text{ZnO}}$)

**Fig. 1:** CGS solar cell energy band diagram of CdS buffer layer with different doping concentrations (a) 10^15^ cm^−3^ (b) 10^16^ cm^−3^ (c)10^17^ cm^−3^ and thickness (10 nm, 50 nm and 100 nm).

The *V*_OC_ of CGS devices is influenced by the built-in electric field and interfacial and bulk recombination. Interfacial recombination and bulk recombination are related to the built-in electric field and external circuit. Therefore, when studying the influence of increasing CdS layer thickness on the *V*_OC_ of the device, it is necessary to consider not only the role of the built-in electric field within the heterojunction but also the influence of external bias on recombination. As the total electric field within the heterojunction weakens under high bias, the role of recombination becomes more significant. Hence, we uniformly investigate the influence of CdS layer thickness on the CdS/CGS heterojunction recombination under a high bias of 0.4 V (near *V*_OC_) to further understand its influence on the *V*_OC_ of the device.

Table 2 and Fig. S2 indicate that when the doping concentration of the CdS layer (10^15^ cm^−3^) is lower than that of the CGS layer (10^16^ cm^−3^), the interfacial recombination (*J*_ifr_) (0.4 V) decreases with an increase in its thickness. This decrease in interfacial recombination (*J*_ifr_) (0.4 V) leads to a decrease in the total recombination (*J*_tot-rec_) (0.4 V), which helps increase the *V*_OC_ of the device. This is consistent with the results shown in Fig. 2a, where the *V*_OC_ increases with an increase in the CdS layer thickness, in the case where the doping concentration of the CdS layer (10^15^ cm^−3^) is lower than that of the CGS layer (10^16^ cm^−3^). When the doping concentration of the CdS layer (10^16^ cm^−3^) is similar to that of the CGS layer, the interfacial recombination (*J*_ifr_) (0.4 V) first decreases (50 nm) and then increases (100 nm) with an increase in its thickness, resulting in a similar trend regarding the total recombination (*J*_tot-rec_) (0.4 V) (Table 2 and Fig. S3). This may explain the observed trend illustrated in Fig. 2a, where the *V*_OC_ first increases (50 nm) and then decreases (100 nm) with an increase in the CdS layer thickness, in the case where the doping concentration of the CdS layer is similar to that of the CGS layer (10^16^ cm^−3^). When the doping concentration of the CdS layer (10^17^ cm^−3^) is higher than that of the CGS layer, the interfacial recombination(*J*_ifr_) (0.4 V) and total recombination (*J*_tot-rec_) (0.4 V) first decrease (50 nm) and then increase (100 nm) with an increase in the thickness of the CdS layer. However, in this case, the *V*_OC_ of the device increases with an increase in the thickness of the CdS layer (Fig. 2a and S4). The reason for the increase in *V*_OC_ may be attributed to the strong built-in electric field (Fig. 1), despite the increase in the heterojunction interfacial recombination (*J*_ifr_)(0.4 V) with a CdS layer thickness of 100 nm.

**Table 2:** The impact of CdS thickness and doping concentration on various recombination currents density at high bias voltage (0.4 V). *J*_tot-rec_, *J*_bulk_, and *J*_ifr_ representing the total recombination current density, bulk recombination current density, and interface recombination current density, respectively.

Doping concentration	Thickness (10 nm)			Thickness (50 nm)			Thickness (100 nm)		
*N*_D_ (cm^−3^)	*J*_tot-rec_ (mA/cm^2^)	*J*_buk_ (mA/cm^2^)	*J*_ifr_ (mA/cm^2^)	*J*_tot-rec_ (mA/cm^2^)	*J*_buk_ (mA/cm^2^)	*J*_ifr_ (mA/cm^2^)	*J*_tot-rec_ (mA/cm^2^)	*J*_buk_ (mA/cm^2^)	*J*_ifr_ (mA/cm^2^)
10^15^	18.1	8.80	9.22	16.8	9.32	7.34	16.4	9.58	6.67
10^16^	19.5	8.62	10.8	18.8	8.37	10.3	22	7.7	14.2
10^17^	24	7.39	16.5	7.63	5.19	2.32	8.43	5.0	3.31

**Fig. 2:** Effect of CdS buffer layer with different doping concentration(10^15^-10^17^ cm^−3^) and thickness (10–100 nm) on the solar cells parameters of CGS solar cells (*N*_A_ ~ 10^16^ cm^−3^). (a) The open-circuit voltage (*V*_OC_), short-circuit current (*J*_SC_), fill factor (*FF*), and efficiency (*E*_ff_).

The aforementioned analysis indicates that when the doping concentration of the CdS layer is confirmed (10^15^–10^17^ cm^−3^), an increase in its thickness to a certain extent (≤50 nm) is beneficial for improving the *V*_OC_ of CGS devices. However, Fig. 2 indicates that the increase in the thickness of the CdS layer is unfavorable for enhancing the performance of CGS devices when the doping concentration of the CdS layer (10^15^ cm^−3^) is lower than or similar to that of the CGS layer (10^16^ cm^−3^). The decrease in *J*_SC_ and fill factor (*FF*) contributes to the decrease in device performance under the aforementioned conditions. First, the weakening of light absorption in the CGS layer caused by the increase in the CdS layer thickness may contribute to the decrease in the *J*_SC_ of the device. Second, Table 3 and Figs. S2 and S3 indicate that when the doping concentration of the CdS layer (10^15^ cm^−3^) is lower than or similar to that of the CGS layer (10^16^ cm^−3^), the increase in the thickness of the CdS layer leads to an increase in interfacial recombination (*J*_ifr_) (0 V) and bulk recombination (*J*_bulk_) (0 V) under short-circuit conditions, which may contribute to the decrease in the *J*_SC_ of the device. The decrease in *FF* caused by the increase in the CdS layer thickness (≤50 nm) (Fig. 2c) is attributed to the increase in *R*_s_ (Figs. S2a and S3a). Figs. S2a–d and S3a–d confirm that the increase in *R*_s_ is associated with the decrease in values of $\frac{\left|\Delta J_{ifr}\right|}{\Delta V}$ near *V*_OC_.

**Table 3:** The impact of CdS thickness and doping concentration on various recombination currents density during short-circuit conditions. *J*_tot-rec_, *J*_bulk_, and *J*_ifr_ representing the total recombination current density, bulk recombination current density, and interface recombination current density, respectively.

Doping concentration	Thickness (10 nm)			Thickness (50 nm)			Thickness (100 nm)		
*N*_D_ (cm^−3^)	*J*_tot-rec_ (mA/cm^2^)	*J*_buk_ (mA/cm^2^)	*J*_ifr_ (mA/cm^2^)	*J*_tot-rec_ (mA/cm^2^)	*J*_buk_ (mA/cm^2^)	*J*_ifr_ (mA/cm^2^)	*J*_tot-rec_ (mA/cm^2^)	*J*_buk_ (mA/cm^2^)	*J*_ifr_ (mA/cm^2^)
10^15^	5.92	5.66	0.15	6.91	6.32	0.47	9.46	6.91	2.44
10^16^	5.82	5.56	0.15	6.17	5.73	0.33	6.18	5.63	0.44
10^17^	5.24	4.85	0.27	5.92	3.79	2.01	6.77	3.67	2.98

When the doping concentration of the CdS layer (10^17^ cm^−3^) is higher than that of the CGS layer, increasing the CdS layer thickness (≤50 nm) becomes beneficial for enhancing the performance of CGS devices. The primary reasons for this improvement include not only the increase in *V*_OC_ but also the enhancement of *FF*. The main factors leading to the increase in *FF* are the increase in *R*_sh_ and the decrease in *R*_s_ (Fig. S4a). The increase in *R*_sh_ is related to the decrease in the values of $\frac{\left|\Delta J_{ifr}\right|}{\Delta V}$ and $\frac{\left|\Delta J_{bulk}\right|}{\Delta V}$ near *J*_SC_ (Figs. 4Sa–d). The decrease in *R*_s_ is associated with the increase in values of $\frac{\left|\Delta J_{ifr}\right|}{\Delta V}$ near *V*_OC_ (Figs. S4a–d).

In summary, for CGS solar cells, when the doping concentration of the CdS layer is lower than or similar to the CGS layer, reducing the CdS layer thickness (such as 10 nm) is beneficial for enhancing the performance of the CGS device. When the doping concentration of the CdS layer is higher than that of the CGS layer, increasing its thickness (such as 30–100 nm) is conducive to improving the performance of the CGS device, and the optimal thickness for maximizing device performance should be approximately 50 nm.

### 3.2 The effect of CdS layer doping concentration on the performance of CGS devices

The aforementioned section demonstrates that the increase in the CdS film thickness can modify the built-in electric field and heterojunction recombination, thereby affecting the device *E*_ff_. This part focuses on the influence of the doping concentration of the CdS layer, with a constant thickness, on the built-in electric field and heterojunction recombination, thereby improving the device performance.

Increasing the doping concentration of the CdS layer is beneficial for enhancing the built-in electric field of the CdS/CGS heterojunction, thus improving the *V*_OC_ of the device. However, as summarized in Table 2 and Fig. S5, when the thickness of the CdS film is 10 nm, an increase in doping concentration can lead to an increase in CdS/CGS heterojunction interfacial recombination (*J*_ifr_)(0.4 V) and total recombination (*J*_tot-rec_)(0.4 V) under high bias, which is unfavorable for improving the *V*_OC_ of the device. Overall, when the thickness of the CdS film is 10 nm, an increase in the doping concentration leads to a slight decrease in the *V*_OC_ of the CGS device (Fig. 2a). Meanwhile, Fig. 2a illustrates that when the thickness of the CdS layer ranges from 30 to 100 nm, the *V*_OC_ of the device first decreases (10^16^ cm^−3^) and then increases (10^17^ cm^−3^), as the doping concentration increases. As the device *E*_ff_ is the highest when the CdS layer thickness is 50 nm, we use it as an example to investigate the influence of doping concentration in the CdS layer on the device parameters. As summarized in Table 2, at a CdS layer thickness of 50 nm, the CdS/CGS heterojunction interfacial recombination (*J*_ifr_)(0.4 V) increases when the doping concentration of the CdS layer increases to a level similar to that of the CGS layer (10^16^ cm^−3^) and decreases when the doping concentration of the CdS layer (10^17^ cm^−3^) increases higher than that of the CGS layer. Therefore, this could be the primary reason why, when the thickness of the CdS layer is within the range of 30–100 nm, as its doping concentration increases, the *V*_OC_ of the device initially declines (when the doping concentration reaches 10^1^⁶ cm⁻³), and subsequently rises (when the doping concentration further increases to 10^1^⁷ cm⁻³).

The aforementioned analysis indicates that an increase in the doping concentration of the CdS layer has varying effects on the *V*_OC_ of the device, depending on the thickness of the CdS layer. However, Fig. 2b–d shows that the increase in the doping concentration of the CdS layer prompts an increase in the *J*_SC_ (except for 100 nm and 10^17^ cm^−3^) and *FF* of the device. Finally, when the thickness of the CdS layer is confirmed (10–100 nm), the increase in its doping concentration helps enhance the performance of the device. The increase in *J*_SC_ with the doping concentration of the CdS layer is associated with a decrease in bulk recombination (*J*_bulk_)(0 V) within the heterojunction under short-circuit conditions (Table 3 and Figs. S5 and S6). Although the *FF* of the device increases with an increase in the doping concentration of the CdS layer, the reasons for this increase vary. According to the I–V curve illustrated in Fig. S5a, when the thickness of the CdS layer is 10 nm, the primary reason for the increase in *FF* with the increase in doping concentration is the decrease in *R*_s_. This decrease in *R*_s_ may be attributed to the increase in $\frac{\left|\Delta J_{Jifr}\right|}{\Delta V}$ near the *V*_OC_ (Figs. S5 a-d). When the thickness of the CdS layer ranges from 30 to 100 nm, the primary reasons for the increase in the *FF* of the device with the increase in doping concentration are the increase in *R*_sh_ and the decrease in *R*_s_. The increase in *R*_sh_ with the increase in the doping concentration of the CdS layer is associated with the decrease in $\frac{\left|\Delta J_{Jifr}\right|}{\Delta V}$ and $\frac{\left|\Delta J_{bulk}\right|}{\Delta V}$ near the *J*_SC_. Simultaneously, the decrease in *R*_s_ is linked to the increase in $\frac{\left|\Delta J_{Jifr}\right|}{\Delta V}$ near the *V*_OC_ (Figs. S6 a-d).

The aforementioned analysis indicated that when the thickness of the CdS layer is thin, such as 10 nm, with an increase in its doping concentration, the improvement in device *E*_ff_ is primarily attributed to the improvement in the *J*_SC_ and *FF*. When the thickness of the CdS layer is thick, such as 30–100 nm, and its doping concentration increases to a level similar to the CGS layer, the enhancement in the *J*_SC_ and *FF* also becomes the primary reason for the improvement in device performance. When the thickness of the CdS layer ranges from 30 to 100 nm and its doping concentration exceeds that of the CGS layer, the *V*_OC_, *J*_SC_, and *FF* of the device considerably improve, and thus, the improvement in device performance is evident.

### 3.3 Comparing with experimental data

We investigate the effects of the thickness and doping concentration of the CdS buffer layer on the performance of wide-gap CIGS solar cells. As wide-gap CIGS solar cells belong to the CIGS solar cell family, adopting their experimental results can approximately verify the rationality of the simulation results. Standard solar cell parameters, including *V*_OC_, *J*_SC_, *FF*, and *E*_ff_, obtained from simulation and experimental data are listed in Table 4, Table 5. The experimental results listed in Table 4 reveal that as the thickness of the CdS layer increases, the CIGS device performance improves (the thickness of CdS layer increases to 50.8 nm), followed by a decline (the thickness of CdS layer increases to 122.9 nm) [30]. The device performance with a thick CdS layer (50.8 and 122.9 nm) is higher than that with a thin CdS layer (32.5 nm). The most appropriate thickness of the CdS layer leading to the optimal device *E*_ff_ of CIGS solar cells is approximately 50 nm. These experimental results are similar to the simulation results obtained with a CdS layer doping concentration of 10^17^ cm^−3^. Meanwhile, the experimental results listed in Table 5 indicate that an increase in the doping concentration of the CdS layer (10^16^–10^17^ cm^−3^), when its thickness is maintained at 50 nm, is beneficial for enhancing the *V*_OC_, *J*_SC_, *FF*, and *E*_ff_ of CIGSSe solar cells [31]. These experimental results are similar to the simulation results as well. Although the experimental and simulation results differ, they exhibit similar trends. Therefore, the simulation results indicate a certain degree of rationality.

**Table 4:** Photovoltaic parameters of CIGS Solar cells with the doping concentration of 10^17^cm^−3^ and various thickness.

Sample	CIGS Thickness (nm)	*V*_OC_ (mV)	*J*_SC_ (mA)	*FF* (%)	*E*_ff_ (%)
Simulated	10	407	17.27	62.94	4.42
	30	558	16.62	65.92	6.11
	50	658	16.59	67.77	7.4
	100	664	15.72	67.48	7.05
Experimental	32.5 [30]	502.1	34.3	47.54	8.19
	50.8 [30]	548.6	37.06	59.98	12.2
	122.9 [30]	545	34.04	61.66	11.44

**Table 5:** Photovoltaic parameters of CIGS Solar cells with the thickness of 50 nm and various doping concentration.

Sample	CIGS doping (#/cm^−3^)	*V*_OC_ (mV)	*J*_SC_ (mA)	*FF* (%)	*E*_ff_ (%)
Simulated	10^15^	528.8	15.6	29.11	2.4
	10^16^	450	16.34	42.74	3.15
	10^17^	658	16.59	67.77	7.4
Experimental	4.84 × 10^16^ [31]	656.3	30.7	67.1	13.52
	2.92 × 10^17^ [31]	676.0	31	68.6	14.3

## 4 Conclusion

This study considered wide-gap CGS solar cells to investigate whether changes in the properties of buffer layers could enhance the built-in electric field of the device and reduce the recombination at the heterojunction interface, thereby improving the *E*_ff_ of CGS solar cells. We selected the most common CdS buffer layer for research. The aim is to determine the optimal parameters of the CdS layer that can enhance the built-in electric field, reduce heterojunction recombination, and improve device performance. This approach can help improve the performance of wide-gap CIGS solar cell devices using other buffer layers (such as Zn(O,S) and Zn(Mg,O)). Our analysis revealed that when the doping concentration of a CdS layer is lower than or similar to a CGS layer, the thickness of the CdS layer that optimizes the performance of the CGS device should be considerably reduced to ensure complete coverage (e.g., 10 nm). However, when the doping concentration of the CdS layer is higher than that of the CGS layer, the optimal thickness of the CdS layer for maximizing the performance of the CGS device should be thicker, for example, 50 nm. Besides the simulation results indicate that the increase in doping concentration of the CdS layer is also beneficial for enhancing the performance of CGS solar cell devices. Especially, when the CdS layer is thicker, such as 50 nm, and its doping concentration increases to higher than that of the CGS layer, the *V*_OC_, *J*_SC_, and *FF* of the device can be simultaneously improved, resulting in a more significant improvement in device performance. In summary, to optimize the performance of wide gap CIGS solar cells, the doping concentration of the CdS layer should be higher than that of the CIGS layer, and its thickness should be approximately 50 nm.

## CRediT authorship contribution statement

**Shiqing Cheng:** Software.

## Declaration of competing interest

We declare that we have no financial and personal relationships with other people or organizations that can inappropriately influence our work, there is no professional or other personal interest that could be construed as influencing the position presented in, or the review of, the manuscript entitled, “*High efficiency wide gap Cu(In,Ga)Se2 solar cells*：*Influence of buffer layer characteristics* ”.
